# Research on Segmenting E-Commerce Customer through an Improved K-Medoids Clustering Algorithm

**DOI:** 10.1155/2022/9930613

**Published:** 2022-06-18

**Authors:** Zengyuan Wu, Lingmin Jin, Jiali Zhao, Lizheng Jing, Liang Chen

**Affiliations:** ^1^College of Economics and Management, China Jiliang University, No. 258, Xueyuan Street, Hangzhou, Zhejiang 310018, China; ^2^College of Optical and Electronic Technology, China Jiliang University, No. 258, Xueyuan Street, Hangzhou, Zhejiang 310018, China

## Abstract

In view of the shortcomings of traditional clustering algorithms in feature selection and clustering effect, an improved Recency, Frequency, and Money (RFM) model is introduced, and an improved K-medoids algorithm is proposed. Above model and algorithm are employed to segment customers of e-commerce. First, traditional RFM model is improved by adding two features of customer consumption behavior. Second, in order to overcome the defect of setting K value artificially in traditional K-medoids algorithm, the Calinski–Harabasz (CH) index is introduced to determine the optimal number of clustering. Meanwhile, K-medoids algorithm is optimized by changing the selection of centroids to avoid the influence of noise and isolated points. Finally, empirical research is done using a dataset from an e-commerce platform. The results show that our improved K-medoids algorithm can improve the efficiency and accuracy of e-commerce customer segmentation.

## 1. Introduction

In recent years, e-commerce has developed vigorously all over the world, with many e-commerce platforms emerging, such as Amazon, Tmall, and JD.com. In 2020, facing the challenges brought by the COVID-19 epidemic to production, operation, and supply chains, e-commerce played an important role in ensuring basic production, supply of living materials, and stimulating economic growth. It is important for e-commerce platforms to gain more customers [1, 2]. In order to gain more customers, they must try to meet the needs of customers [3, 4]. Different customers need different services and products, leading to the diversification of customer needs [5]. Customers segmentation is the basis of analyzing the diverse needs of different customers. Customer segmentation is to subdivide customers with different attributes and features into specific categories, which is an important tool to effectively identify the value of customers, and it can help online merchants to develop personalized marketing strategies for customers of different value categories [6–8]. Customer segmentation enables platforms to become more client centric [9]. Only with an in-depth understanding of the preferences and needs of different customer groups, precision marketing can be implemented.

In the field of customer segmentation, RFM is most classical model, which is proposed by Hughes [10]. On the base of RFM model, many scholars developed clustering analysis technique to segment customers [11]. However, there are still some gaps in the existing literature. First, in terms of feature selection, the existing literature focused on using the historical order data of customers, which cannot fully reflect the behavioral preferences and consumption habits of different customer groups. Second, in terms of selecting cluster algorithm, the K-means clustering algorithm proposed by the existing literature did not consider the algorithm operation efficiency.

Based on the above considerations, in this article, we study strategies for optimizing clustering algorithms to improve the performance of e-commerce customer segmentation. We made some improvements in feature selection and clustering algorithms. First, when selecting features, we introduce customer consumption behavior data into the traditional RFM model, including data added to shopping cart (C) and favorites (V). Second, in terms of algorithm improvement, we address the problem of artificially setting *K* values in the K-medoids algorithm and introduce the CH as clustering quality evaluation index to determine the best *K* values. Meanwhile, according to the problem that the K-medoids algorithm is sensitive to the initial clustering center, we combine the K-means++ algorithm to improve the selection of clustering center. The experimental results show that the improved K-medoids algorithm can effectively alleviate the sensitivity of the algorithm to noise and initial clustering center selection. The algorithm also considers the operational performance of the algorithm, so as to improve the efficiency and accuracy of e-commerce customer segmentation.

The rest of this paper is organized as follows. In Section 2, the existing literatures on customer segmentation are reviewed and the research gaps are proposed. In Section 3, the improved K-medoids algorithm is described in detail. In Section 4, empirical research is done using an e-commerce dataset and the empirical results are analyzed. In Section 5, the contributions, shortcomings, and future research are discussed. Finally, the conclusions are drawn in Section 6.

## 2. Literature Review

Existing literature on customer segmentation is divided into two fields. The first is about selecting different segmentation features. The second is about selecting and improving the clustering algorithms. In terms of the selection of segmentation features, the existing literature can be divided into three types from different perspectives [12], including demographic perspective, customer life cycle perspective, and customer behavior perspective. Firstly, scholars [13] who conducted research from the perspective of demography mainly collected data using questionnaire surveys. They divide customers into different groups according to their age, gender, family income, marital status, education, etc. Secondly, literature studying this issue from the perspective of the customer life cycle [14] divides the customer life cycle into several stages according to the number of new customers, retained customers, and lost customers. In different stages, companies should take different measures for them. The customer loyalty classification method [15, 16] is the most popular segmentation method in existing segmentation literature. Third, with the continuous development of data mining technology, the indicator selection methods based on customer behavior are becoming a hot topic. In these literatures, multidimensional features are used to reflect the consumption behaviors and habits of different customer groups [17, 18]. As a classic customer value model, the RFM model has been successfully applied to customer segmentation [19, 20]. Due to features in different industries, some scholars have improved and extended the RFM model [21–24]. However, the consumer behavior preference among different customer groups cannot be well identified. Yoseph et al. [25] studied consumer behavior (e.g., clicking on product links, browsing products, and adding to cart) and purchasing power, and added these features to the RFM model so that consumer categories could be accurately identified and differentiated.

K-means algorithm and K-medoids algorithm are the most commonly used clustering algorithms. K-means has been widely applied in the fields of data mining and pattern recognition because of its advantages such as simple operation and fast speed. However, the traditional K-means algorithm is susceptible to noise and isolated points, which leads to poor clustering results [26]. K-medoids algorithm is another classical division-based clustering method [27]. Compared with K-means, this algorithm optimizes the selection method of the center of mass, overcomes the defect of being sensitive to isolated points, and has higher clustering accuracy. However, the K-medoids algorithm still has the problem of being vulnerable to the initial clustering center. To address the above problem, many scholars have proposed a series of improved algorithms for K-medoids.

According to the problem of the selection of initial clustering centers, two improvement ideas are mainly proposed in existing literature. First, based on the K-medoids algorithm, existing literatures optimize the selection of initial clustering centers using the distance or correlation between samples [28, 29]. This improved method is based on the following principle. Since the cluster centers are usually the more important sample points in a cluster, the denser the sample points are with strong correlation with other sample points, the easier they are to become the best cluster centers. Ho-Kieu et al. [28] proposed an improved initial center selection method by introducing probability density function. The experimental results showed that the improved algorithm had obvious advantages compared with the original K-medoids algorithm. The above improved methods optimize K-medoids for the selection of initial clustering centers, reduce the number of iterations, and improve the clustering efficiency. However, these selection methods only consider the distance or correlation between samples, which is easy to make the clustering results fall into local optimum. They cannot achieve more accurate clustering results for datasets with large disparity in the number of samples between clusters.

Second, some scholars introduce the Swarm Intelligence [30, 31] and combine it with K-medoids to improve the global search capability and efficiency of the improved algorithms for samples. Arthur and Vassilvitskii [32] algorithmically fused the Swarm Algorithm with K-medoids. The experimental results showed that the improved algorithm effectively reduced the influence of noise on the clustering results and improved the clustering accuracy. This type of improved algorithm effectively avoids the problem of local optimum of clustering results. However, it is worth noting that the integration with the Swarm Intelligence will lead to the increase in algorithm complexity and the reduction in operation efficiency. The huge transaction volume and mass data in e-commerce platforms require high clustering efficiency. It is necessary for platform managers to segment customer timely in order to manage e-commerce customers well. Therefore, we try to solve the problem of sensitivity to the initial clustering center that exist in K-medoids algorithm while ensuring the operational efficiency of the algorithm in this paper.

In summary, in existing e-commerce customer segmentation literature, there are still two gaps that have not been solved well. First, from the perspective of selecting segmentation features, the existing literatures focus on using the historical order data of customers. But the consumption behavior data of customers is ignored, which cannot more comprehensively reflect the behavioral preferences and consumption habits of customers in different customer groups. Second, from the perspective of clustering algorithms, although the improved K-medoids algorithm in existing literature alleviates the sensitivity of the algorithm to the initial clustering center and improves the clustering performance, there are still limitations in the two aspects. First, the clustering results may fall into the local optimum. Second, the algorithm may run less efficiently.

Therefore, we attempt to solve the above problems. First, while selecting segmentation features, we construct a new model by incorporating customers' online consumption behavior, where Recency, Frequency, Money, Add to Cart, and Add Favorites are included. For clarity, this model is called a RFMCV model. Second, considering the defect of artificially set K values in the K-medoids algorithm, we introduce the CH index to determine the best K values. Third, drawing on the idea of K-means++ algorithm [33] for selecting initial clustering center, the K-medoids algorithm is improved. Finally, the algorithm proposed in this paper is validated on two standard test datasets.

## 3. Improved K-Medoids Algorithm

In this paper, we improve K-medoids algorithm from two aspects. First, the CH evaluation index is introduced in order to determine the optimal number of clusters in the K-medoids algorithm. Second, the idea of K-means++ algorithm is introduced while selecting initial clustering centers.

### 3.1. Description of the K-Medoids Algorithm

Both K-means and K-medoids algorithms are classical division-based clustering methods, which generally use Euclidean distance as a measure of similarity between two data points. The smaller the distance, the greater the similarity. However, the K-medoids algorithm is optimized for the selection of centroids to avoid the influence of noise and isolated points [34]. The algorithm is implemented in the following steps. First, input dataset and the number of clusters. Second, initialize the clustering centers and assign samples. Randomly select the initial clustering centers, calculate the Euclidean distance between the remaining data points and the clustering center, find the shortest distance, and assign all samples to the clusters corresponding to the clustering center. Third, update the cluster centroids. Randomly select a noncentroid, and replace the clustering centers according to the principle of squared error function value reduction. Finally, iterative calculation is performed until the clustering center no longer changes or the maximum number of iterations is reached. Then, the cycle ends and the final clustering result is obtained.

### 3.2. Implementation Procedure of the Improved K-Medoids Algorithm

### 3.3. Determine the Optimal Number of Clusters *k*

We introduce the CH clustering quality evaluation index [32] and set the class corresponding to the highest CH value as the number of clusters. The CH value is the ratio of intercluster sample separation to intracluster sample tightness, and a larger CH represents a tighter class itself and a more dispersed class to class (i.e., a better clustering result). When the intracluster is dense and the intercluster separation is good, the optimal number of clusters can be clearly derived from the CH value line graph, and it has the advantage of fast calculation speed.

The calculation formula of CH value is as follows.

(1) $$\begin{array}{c} S\left(k\right)=\left(\frac{\text{BGSS}}{\text{WGSS}}\right)\times \left(\frac{m-k}{k-1}\right). \end{array}$$

Within-Groups Sum of Squared Error (WGSS) is the sum of squared errors within clusters. It is used to measure the tightness of samples within clusters. The smaller the WGSS is, the tighter the clusters are and the better the clustering effect is. Its calculation formula is

(2) $$\begin{array}{c} \text{WGSS}=\frac{1}{2}\left[\left(m_{1}-1\right)\bar{d_{1}^{2}}+\cdots +\left(m_{k}-1\right)\bar{d_{k}^{2}}\right], \end{array}$$

where $\bar{d_{1}^{2}}$ is the average distance of samples within the *k*-th cluster; *m*_*k*_ is the number of samples in the *k*-th cluster.

Between-Groups Sum of Squared Error (BGSS) is the sum of squared errors between clusters, which is used to measure the separation of samples between clusters. The larger the BGSS is, the more dispersed the clusters are and the better the clustering effect is. Its calculation formula is

(3) $$\begin{array}{c} \text{BGSS}=\frac{1}{2}\left[\left(k-1\right)\bar{d^{2}}+\cdots +\sum_{j=1}^{k}\left(m_{j}-1\right)\left(\bar{d^{2}}-\bar{d_{j}^{2}}\right)\right], \end{array}$$

where $\bar{d^{2}}$ is the average distance between all samples, $\bar{d_{j}^{2}}$ is the average distance of samples within the *j*-th cluster, *m*_*j*_ is the number of samples in the *j*-th cluster, and *k* is the number of sample clusters.

### 3.4. Comparison and Validation

In order to verify the effectiveness of the improved K-medoids proposed in this paper, two comparison experiments are conducted. First, we compare the performance of clustering algorithms. Second, we compare the clustering quality evaluation indicators.

#### 3.4.1. Comparison of Algorithm Performance

In order to verify the effectiveness of the algorithm, two standard test datasets were selected for the experiments, including breast cancer [35] and iris plants [36] in UCI database. UCI database is the most popular dataset in the field of machine learning, which is built by University of California Irvine. Furthermore, K-medoids, K-means++, and spectral clustering (SC) method were selected to compare with the improved K-medoids algorithm proposed in this paper. Both the clustering accuracy and the running time of 4 algorithms on the two datasets were mainly compared. The results are shown in Table 1.

As can be seen from Table 1, the improved K-medoids algorithm has an accuracy of 86.8% on the breast cancer dataset, outperforming the K-medoids, K-means++, and spectral clustering methods in terms of clustering accuracy. Meanwhile, the running time of the improved K-medoids algorithm is shorter than the other 3 algorithms, which is 22.7 ms. On the iris plants dataset, the improved K-medoids algorithm has the highest accuracy of 84% and the shortest running time of 13.9 ms. Therefore, among the four algorithms, the improved K-medoids algorithm has the best performance in terms of accuracy and clustering efficiency. Based on the above analysis, the improved K-medoids algorithm proposed in this paper outperforms the other three clustering methods on both datasets.

#### 3.4.2. Comparison of Clustering Quality Evaluation Indicators

In order to determine the best K value, the CH index is introduced to decide the K value in this paper. In order to verify the applicability of the CH index for customer segmentation in the e-commerce industry, we use the e-commerce dataset in practice. Furthermore, the result is compared with the inflection point method. The experimental result of CH value is shown in Figure 1. The experimental result of the inflection point method is shown in Figure 2.

As can be seen from Figure 1, the line chart of CH value shows a line rising and then falling trend, and the highest CH value is obtained when the number of clusters is 4. Therefore, using the CH index, it can be clearly concluded that the optimal number of clusters for this e-commerce platform dataset is 4.

The principle of the inflection point method is to obtain the optimal number of clusters at the inflection point of the line graph, because continuing to increase the K value after the inflection point does not increase the classification accuracy much, but increases the number of clusters. In Figure 2, the horizontal axis is the number of clusters, and the vertical axis is the sum of squares due to error (SSE). As can be seen in Figure 2, when the K value changes from 4 to 19, the change in the folding graph is smoother (i.e., there is no obvious inflection point to accurately determine the optimal number of clusters).

The above analysis shows that the CH index is better than the inflection point method in the segmentation of e-commerce customers.

## 4. Empirical Analysis

### 4.1. Selecting Features for Customer Segmentation

RFM model was first proposed by Hughes [10], which is generally an analysis tool used to identify an organization's best customers. RFM model is based on 3 factors, including Recency (*R*), Frequency (*F*), and Monetary value (*M*). Recency (*R*) usually represents how recently a customer has made a purchase. The more recently a customer has made, the more likely he will continue to keep the relationship. Frequency (*F*) usually represents how often a customer makes a purchase within the observation period. The larger the *F*-value represents the idea that the more frequent the customer consumption, the higher the customer value. Monetary (*M*) usually represents how much money a customer spends on purchases within the observation period. The larger the *M*-value, the higher the customer value. Since its introduction, the RFM model has been widely used in customer segmentation [29].

The traditional RFM model has been widely used for customer segmentation in various industries. However, there are still several problems. The RFM model cannot reflect the customer's activity on the e-commerce platform and the differences in consumption and behavior between different customer groups. With the development of big data technology, the dimensions of customer data extracted from e-commerce platforms are increasing, and these data reflect customers' value characteristics, consumption habits, and behavioral preferences in a more detailed and comprehensive way. Therefore, based on the traditional RFM model, we integrated customers' online behavioral indicators and proposed the RFMCV model for e-commerce customer segmentation, in which C and V indicators could reflect customers' s activity and online consumption habits. Add to cart (C) represents frequency that a consumer has added a product to their shopping cart. Add favorites (V) represents the frequency that a consumer has added a product to their product favorites. Both of these behaviors represent the consumer's preference for a product. The higher the frequency is, the more likely consumers are to buy the product. The introduction of these two indicators into the RFM model can effectively improve the effectiveness of the RFM model for e-commerce customer segmentation [25].

### 4.2. Data Description

The customer consumption data in this paper is from Kaggle database [37]. There are 100,000 orders from multiple marketplaces in Brazil from 2016 to 2018. Many features are contained in this dataset, including order status, price, payment, and freight performance to customer location, product attributes, and reviews written by customers. Then the order and online behavior data of 37,376 customers were extracted from this dataset. The consumption time is from November 18, 2017, to December 18, 2017. In order to segment e-commerce customers, we select 5 fields. The fields and descriptions in the dataset involved in this dataset are shown in Table 2.

### 4.3. Data Preprocessing

#### 4.3.1. Data Cleaning

The behavioral data of these e-commerce customers in a month is about 100,000 pieces, and data cleaning is needed. Firstly, data with missing and abnormal values are processed, such as data with zero expense, data with purchase date as the idle value, and data with obviously wrong expense. Secondly, duplicate data are processed. The user's purchase behavior is accurate to the hour. There will be a small number of users who repeatedly purchase or add favorites within an hour, so this kind of data will be processed. Finally, the consistency of the data is dealt with. The indicator *R* involves time features. The date and hour in the time data exist in one field, so it is split into two fields. In addition, we convert the field type in the Timestamp field into the form of year, month, and day to facilitate the calculation of time.

#### 4.3.2. Indicator Extraction and Normalization

The individual indicators in the RFMCV model are explained in detail as follows:

 
*R*: recency: the time interval between the customer's last purchase in the observation period and 31 December 2017.
 
*F*: frequency of customer purchasing in the observation period.
 
*M*: monetary: the amount spent by the customer in the observation period.
 
*C*: frequency of the customer who added the product to cart in the observation period.
 
*V*: frequency of the customer who added the product to favorites in the observation period.

According to the RFMCV model proposed in this paper, 37,376 samples are collected, and some of them are shown in Table 3.

In order to avoid the disparity caused by the different units of each indicator, the dataset after indicator extraction needs to be normalized prior to experimental analysis. The *Z*-score normalization method is employed in this paper, which normalizes the data by giving the mean and standard deviation of the original data. The processed data yields the standard normal distribution (i.e., the mean value is 0 and the standard deviation is 1). The transformation function is

(4) $$\begin{array}{c} X^{*}=\frac{X-\mu }{\sigma }, \end{array}$$

where *μ* is the mean of all samples and *σ* is the standard deviation of all samples.

After the normalization process, all data were converted to dimensionless data. Partial data is shown in Table 4.

### 4.4. Analysis of Empirical Results

According to the experimental results in Section 3.2, the optimal number of clusters *k* is 4. Based on the RFMCV model, the improved K-medoids algorithm is run. The results show that all customers are divided into 4 groups, named Type A, Type B, Type C, and Type D. The distribution of each indicator of the RFMCV model of four customer types is shown in Figure 3.

Comparing the customer indicators of each group among the 4 groups in Figure 3, some findings can be drawn.

The value of Type B customers is the highest, which includes 13,415 customers, accounting for 35.89% of total e-commerce customers. *R*-value of the Type B customers is smaller; their last purchase on this platform is more recent. The *F*-value is the highest, suggesting that the frequency is high and that they are active customers on this e-commerce platform. *M*-value is the biggest; they spend the most in this platform. *C*-value is the biggest; they add to cart most frequently. However, *V*-value is small, which shows that these customers often add to cart rather than add favorites when they find interesting products. This group has the highest current value and value-added potential and should be classified as a high-value customer group in this e-commerce platform. For this group, platform owners should put significant effort and resources into maintaining and developing good relationships with them. Effective measures should be taken to tap their consumption potential.

The second valuable customer group is type A, which includes 7,463 customers, accounting for 19.97% of total customers. *R*-value of the Type A customers is smaller than Type B and Type D, and they make a purchase most recently. Both *F*-value and *M*-value of Type A are the second biggest among the 4 groups. They are more active customers and spend more on this e-commerce platform. Different from Type B, *C*-value of these customers is low, but the *V*-value is the highest among these four groups. It shows that these customers are used to adding favorites when they find interesting products. According to the above analysis, customers of Type A can be classified as the second valuable group. These customers have greater potential for value mining. The platform owners should hold some promotional activities in order to stimulate their consumption potential.

The third customer group is Type D, which includes 14,340 customers, accounting for 38.37% of total e-commerce customers. These customers have the biggest *R*-value, indicating that they have not purchased goods from this platform for a long time. *F*-value, *M*-value, *C*-value, and *V*-value are all small, indicating that this group of customers is inactive in this e-commerce platform. They do not frequently add favorites or add to cart on the platform. They can be classified as a low-value customer group. However, the number of this group is big, and their consumption frequency is medium. It is necessary for platform owners to enhance the value of this group by personalized push products.

The fourth customer group is Type C, including 2,158 customers, accounting for 5.77% of total e-commerce customers. *R*-value of this customer group is low, and *F*-value is smallest, indicating that this group has recently spent money on the platform, but the overall consumption frequency is low. *M*-value, *C*-value, and *V*-value are smallest; they are also inactive customers. Unlike those customers of Type D, they complete their last purchase at a very close time, so they are likely to be new customers. Special attention needs to be paid to them. It is important to understand their needs and develop good relationship with them.

## 5. Discussion

The main contributions of this paper are the following. Firstly, this research enriches the theoretical research related to customer segmentation. The research object of this paper is e-commerce customers, whose consumption behaviors are based on the Internet platform. It is necessary to add more new online characteristics and consumption patterns. Therefore, we integrate two features of online consumption behavior into RFM model, including adding to cart (C) and add favorites (V). Secondly, in order to solve the problems of artificially setting *K* values and sensitivity to the initial clustering centers, we improve the existing K-medoids clustering algorithm by introducing CH cluster quality evaluation index and idea of K-means++ algorithm. Furthermore, data from both simulated dataset and the real dataset are used to test the performance of improved K-medoids. In practice, the findings in this paper will enable e-commerce platforms to identify different kinds of customers. According to different kinds of customers, different preventive measures can be taken. It will help to maintain the important profit source for an e-commerce platform, thus achieving a “win-win” situation for both platforms and consumers.

## 6. Conclusion

It is necessary for an e-commerce platform to segment customers before implementing a marketing strategy. In other words, customer segmentation is the base of accurate marketing. In the era of big data, machine learning is an important tool which can help platforms to analyze consumption behavior. In view of some gaps in the existing literature, some improvements have been made in this paper. First, we improve the traditional RFM model by integrating the consumption behavior of customers. Second, the CH index is introduced to determine the best K value. Third, combining with the K-means++ algorithm, the K-medoids algorithm is improved by optimally selecting the initial clustering center. Finally, an empirical analysis was conducted using a sample of 37,376 customers from an e-commerce platform.

Based on the comparison with other algorithms and empirical analysis, three conclusions can be drawn. First, the RFMCV model proposed in this paper is an effective index system to segment customers. The five features selected in this model integrated customer value features and customer consumption behavior features, which can be used to distinguish different consumption habits and preferences. Second, compared with the inflection point method, the CH index introduced in this paper is more suitable for e-commerce datasets. Third, compared with the K-medoids algorithm, K-means++ algorithm, and spectral clustering method, the improved K-medoids algorithm proposed in this paper can gain better clustering accuracy and efficiency.

However, there are still some potential limitations in this paper, and some future research can be done. First, we introduce two features C and V into the RFM model to improve the accuracy of e-commerce customer classification. In the future, more features of consumer behavior (e.g., clicks, comments, etc.) can be integrated into the model to classify customers. Second, we improve K-Medoids algorithm for clustering in this paper. We verify the effectiveness of our improved K-medoids algorithm using two standard test datasets, and then employ this algorithm to segment e-commerce customers. In future research, we will use hierarchical clustering, density-based clustering and other methods to cluster e-commerce customers. Furthermore, we plan to compare the clustering performance of these methods with that of K-Medoids. Third, the available data in this paper could be affected by uncertainties or inaccuracies. In view of this problem, some scholars put forward solutions. Versaci et al. [38] proposed a new approach to assess the mechanical integrity of a steel plate, which translated this problem into a classification problem by using fuzzy similarity computations. In order to handle the data uncertainty, Ontiveros-Robles and Melin [39] proposed a specific kind of computer-aided diagnosis system based on General Type-2 Fuzzy Logic. In the future, it would be necessary to use fuzzy classification systems.

In this paper, we improve the RFM model by introducing customer's behavioral features, and employ an improved clustering algorithm to segment e-commerce customers. Firms can improve the effectiveness of customer segmentation by using our proposed model. In addition, they can understand the needs of different customers, which helps promote the innovation of enterprises from the source.

## Figures and Tables

**Figure 1:** Line chart of CH value.

**Figure 2:** Line chart of inflection point method.

**Figure 3:** Distribution chart of four groups.

**Algorithm 1:** Implementation procedure of the improved K-medoids algorithm.

**Table 1:** The performance of 4 algorithms working on different datasets.

Datasets				
Clustering algorithm	Breast cancer		Iris plants	
	ACC (%)	Time (ms)	ACC (%)	Time (ms)
K-medoids	0.858	33.1	0.663	26.5
K-means++	0.854	208.2	0.833	265.0
Spectral clustering	0.667	103.8	0.9	118.1
Improved K-medoids	0.868	22.7	0.840	13.9

**Table 2:** The fields and descriptions in the dataset.

Field name	Data type	Field description
Customer_unique_id	Int	Customer's unique identification
Order_id	Int	Order identification
Product_id	Int	Product identification
Behavior type	String	The type of user behavior towards the product, including browsing, favoriting, adding to cart, purchasing
Timestamp	Int	Time of behavior

**Table 3:** Partial data of RFMCV model.

Customer_unique_id	*R*	*F*	*M*	*C*	*V*
5	1	1	99	13	7
18	6	2	210	16	0
22	4	8	84	0	0
…	…	…	…	…	…
906311	7	5	118	7	0
906338	3	1	28	5	0
906355	5	4	84	9	0

**Table 4:** The table of partial data of RFMCV model after normalized treatment.

Customer_unique_id	*R*	*F*	*M*	*C*	*V*
5	−0.000902	2.068466	−0.097700	−0.745080	−0.397498
18	−0.623415	−0.018191	1.465430	1.340590	−0.390554
22	1.247733	3.807347	0.597041	−0.390554	−0.390554
…	…	…	…	…	…
906311	−0.625219	−0.365967	−1.139736	−0.397498	−0.390554
906338	0.935574	1.025137	0.324119	0.167400	−0.390554
906355	0.311257	−0.677361	−0.097700	0.428109	−0.390554

## Data Availability

The data used to support the findings of this study are available from the UCI repository “Breast Cancer Data Set” and “Iris Data Set”, and the Kaggle repository “Brazilian E-Commerce Public Dataset by Olist.”
